The article "TCM Constitution Analysis Method Based on Parallel FP-Growth Algorithm in Hadoop Framework" was published in 2022. Journal: J Healthc Eng.

# TCM Constitution Analysis Method Based on Parallel FP-Growth Algorithm in Hadoop Framework

**DOI:** 10.1155/2022/9006096

**Published:** 2022-08-30

**Authors:** Mingzheng Li, Xiaojuan Lv, Ye Liu, Lin Wang, Jianqiang Song

**Affiliations:** ^1^School of Information Engineering, Henan University of Science and Technology, Luoyang 471003, China; ^2^Lushi Chinese Medicine Hospital, Lushi County, Sanmenxia 472100, China; ^3^Information Department of PLA Rocket Force Characteristic Medical Center, Beijing 100120, China; ^4^Henan Qunzhi Information Technology Co. Ltd., Luoyang 471003, China

## Abstract

This work is devoted to establishing a comparatively accurate classification model between symptoms, constitutions, and regimens for traditional Chinese medicine (TCM) constitution analysis to provide preliminary screening and decision support for clinical diagnosis. However, for the analysis of massive distributed medical data in a cloud platform, the traditional data mining methods have the problems of low mining efficiency and large memory consumption, and long tuning time, an association rules method for TCM constitution analysis (ARA-TCM) is proposed that based on FP-growth algorithm and the open-source distributed file system in Hadoop framework (HDFS) to make full use of its powerful parallel processing capability. Firstly, the proposed method was used to explore the association rules between the 9 kinds of TCM constitutions and symptoms, as well as the regimen treatment plans, so as to discover the rules of typical clinical symptoms and treatment rules of different constitutions and to conduct an evidence-based medical evaluation of TCM effects in constitution-related chronic disease health management. Secondly, experiments were applied on a self-built TCM clinical records database with a total of 30,071 entries and it is found that the top three constitutions are mid constitution (42.3%), hot and humid constitution (31.3%), and inherited special constitution (26.2%), respectively. What is more, there are obvious promotions in the precision and recall rate compared with the Apriori algorithm, which indicates that the proposed method is suitable for the classification of TCM constitutions. This work is mainly focused on uncovering the rules of “disease symptoms constitution regimen” in TCM medical records, but tongue image and pulse signal are also very important to TCM constitution analysis. Therefore, this additional information should be considered into further studies to be more in line with the actual clinical needs.

## 1. Introduction

The diagnosis and treatment methods of TCM are the crystallization of the wisdom of the Chinese nation over thousands of years, and the precious wealth of the TCM industry and the world health system. Guided by the worldview and methodology of ancient Chinese philosophy, TCM carries the experience and theoretical knowledge of Chinese people's struggle against diseases, forming a holistic medical system through long-term practice and accumulating amount of clinical data. Meanwhile, TCM has played an extremely important role in the prevention and control of major infectious diseases in New China. Especially, it is proved once again that TCM is a treasure to protect people's health and lives to combat COVID-19 since 2019 [1]. A lot of studies based on machine learning and image processing have been implemented on the informatization and wisdom of TCM. Among them, the theory of TCM constitution is of great guiding significance for disease prevention and therapy. Based on the results of TCM constitution analysis in different populations, combined with their geographical and climate environments, targeted regimens or treatments are developed to carry out early health intervention or disease control to promote people's immunity and alleviate patients' symptoms, which is also important to reduce the incidence of COVID-19 and speed up the cure of patients.

The article "TCM Constitution Analysis Method Based on Parallel FP-Growth Algorithm in Hadoop Framework" was published in 2022. Journal: J Healthc Eng.

TCM has paid great attention to individual syndrome differentiation. In the theoretical system of TCM, the constitution of the Chinese people is divided into nine types, namely, balanced constitution (BC), yang-deficiency constitution (YADC), yin-deficiency constitution (YIDC), qi-deficiency constitution (QDC), qi-stagnation constitution (QSC), phlegm-dampness constitution (PDC), dampness-heat constitution (DHC), blood stasis constitution (BSC), and inherited special constitution (ISC). Each physique has a series of different health preserving and conditioning programs including diets, sports, meridians, and so on. Therefore, the conditioning program should be recommended according to the current specific physical state. For example, yang-deficiency constitution is mainly characterized by fear of cold, pale face, fatigue, and cold body. So, the patients with yang-deficiency constitution are usually advised to keep warm, such as warm diet, special acupoints (such as Qihai, Zusanli, Yongquan, and Shenque) massage, more exercise, and so on. Yin-deficiency constitution is mainly characterized by fear of hot, dry mouth and throat, hot hands and feet, so the patients with yin-deficiency constitution are normally advised to pay special attention to their lungs and kidneys, such as eating more nourishing and refreshing food, and avoiding that makes ones feel hot and dry. Similarly, the other seven constitutions also have their own unique health conditioning programs.

The article "TCM Constitution Analysis Method Based on Parallel FP-Growth Algorithm in Hadoop Framework" was published in 2022. Journal: J Healthc Eng.

TCM constitution analysis takes people's constitution as the cognitive object and tried to grasp the overall elements of individual health and disease according to the characteristics of different constitutions to formulate a unique prevention and treatment principle, grasping the overall elements of individual health and disease differences from the characteristics of different constitution to formulate the principle of prevention and treatment. Therefore, its automation has become a research hotspot in modern Chinese medicine. TCM constitution automatic analysis is a very practical application for the exploration of TCM standardization. Modern Chinese medicine constitution analysis system combines Internet and artificial intelligence technologies, adopts deep learning model and backpropagation algorithm and data mining methods to extract TCM constitution features from the fused multimodal data that derived from tongue, face, plus diagnoses and so on, and dig out the correlations between syndrome, regimen, and constitution to realize TCM constitution automatic analysis.

However, the TCM constitution is still faced with severe challenges due to the lack of knowledge model and objective evaluation criteria with normative diagnosis and treatment mode, which makes it difficult to adapt to the current “Internet +” diagnosis and treatment mode. For example, the existing TCM constitution analysis systems on the market only provide a personal report with some simple food therapy, exercise, and recuperation information, which is lack of the correction between symptoms and prescriptions. Fortunately, modern computer technology brings light on new research ways of upgrading TCM constitution analysis. One effective method that has been widely used in the TCM constitution field is data mining, which is used to extract useful, hidden, and unknown inner connections and knowledge from a large number of TCM clinical records stored in an electronic database to discover the rules implicit in data and predict future trends of TCM diagnosis and treatment [2, 3].

Data mining techniques (association rule mining, Classification, clustering, etc.) have been widely used in the field of health care, such as heart disease diagnosis [4], DNA patterns recognition [5, 6], ultrasound image segmentation [7, 8] and so on, which is aiming to dig out the valuable correlation implicit in a large amount of data [9–11]. Among them, association rule algorithms are usually used to discover the interdependence and relevance between symptoms, differentiation, diagnosis, and prescription for treatment of diseases. For example, Fengxia [12] tried to explore the relationships between “principle-prescription-herbs” in the diagnosis of liver diseases through association rules. Kennedy and Carrazza [13] made a quantitative analysis of the correlation between relevant semantic features in the pulmonary nodules database by setting the standards of support and confidence in association rules, and further improved the ability of clinical radiologists to detect and diagnose pulmonary nodules by setting new evaluation indexes for the importance of individual features.

The article "TCM Constitution Analysis Method Based on Parallel FP-Growth Algorithm in Hadoop Framework" was published in 2022. Journal: J Healthc Eng.

In recent years, association rule algorithms have also been used in the field of TCM and achieved many gratifying research results. For instance, Yadong et al. [14] used Apriori algorithm to study the relations between drugs' dose and lung-cancer patients' responses and analyzed the proportional relationship between the dosages of different drugs to provide a reference for clinical doctors. Chen et al. [15] investigated the efficiency in TCM dispensing based on the frequent pattern (FP) growth algorithm and tried to identify which 2 or 3 herbal medicines will match together frequently in prescriptions. Yang et al. [16] used Apriori algorithm to explore the association rules of breast cancer and TCM syndrome to provide effective treatment for patients. Leem et al. [17] used association rule mining and network to analyze the combinations of medicinal herbs used to treat alopecia and identified frequently combined two-herb and three-herb sets. These achievements have provided auxiliary references for TCM constitution automatic analysis to a certain extent. As it is well known that FP-growth method only needs to scan the entire database twice without generating a large number of candidate frequent sets, which makes it faster than Apriori algorithm and usually two orders of magnitude better speed performance [18, 19]. Usually, FP-growth algorithm adopts the following dip-and rule strategy to produce frequent item sets more efficiently by compressing the frequent item sets into an FP-tree and can still retain the association information of frequent items.

In this work, a TCM constitution automatic analysis method (ARA-TCM) based on FP-growth algorithm in the Hadoop framework is proposed, which is used to establish a comparatively accurate classification model between the 9 kinds of constitutions and their typical clinical symptoms and treatment plans. Then the experiments were applied to a self-built medical database with 30,071 pieces of records and the results have demonstrated several advantages as follows: Firstly, dozens of medical laws for each physical constitution have been excavated to build an association rule library of “disease symptoms constitution regimen” to provide preliminary screening and decision support for TCM clinical health management. Secondly, new treatment rules for chronic disease and new combinations of TCM herbs appeared in the mined rules, which will have a certain promoting effect on the study of Chinese medicine tablets. Finally, the proposed method has shortened the overall cluster working response time and has higher computational efficiency, precision, and recall rates compared with the traditional Apriori and FP-growth algorithms at the same time.

The article "TCM Constitution Analysis Method Based on Parallel FP-Growth Algorithm in Hadoop Framework" was published in 2022. Journal: J Healthc Eng.

The rest of the article is organized as follows: Section 2 surveys the related work about the proposed method.  Section 3 elaborates the whole framework of the proposed method.  Section 4 describes the proposed method in detail and presents the experiments and evaluates the results. Finally, some conclusions are given in Section 5.

## 2. Related Work

### 2.1. FP-Growth Algorithm

Compared with Apriori algorithm, FP-growth algorithm uses a clever and compact data structure called FP-tree to extract frequent item sets directly and reduce the time and operation cost, avoiding scanning the whole database and generating the candidate frequent item queue constantly. It only needs to scan the whole transaction database twice to get a frequent 1-item set and create an FP-tree, respectively. The main idea of FP-growth algorithm is to map every transaction in the database into an FP- tree and retain the association information between the item sets at the same time. The primary task of data mining with FP-growth algorithm is to construct a header table to construct the conditional FP-tree. The compressed database is divided into a set of conditional databases to be associated with a frequent item or a pattern segment. After creating the root node, each transaction in the database is processed as follows to generate an FP-tree to mine the frequent item set recursively. The whole framework of FP-growth algorithm is shown in Figure 1.

The process of constructing an FP-tree is described as follows:

- Build a frequent item list *F*_list._
- At first, scan the entire database and count the frequency of each data item to filter out the data items with a lower frequency than the minimum support threshold, and then sort all the rest of the data items in the order of decreasing frequency to obtain *F*_list_.
- Create the FP-tree.
- Firstly, sort each transaction according to the position of data item in *F*_list_, and get rid of the transaction that corresponds to the data item with a low frequency less than the minimum support degree; Secondly, insert the sorted transactions into the prefix tree and record the frequent number of the shared tree nodes with a common prefix, which is used to represent the number of occurrences of each node. To facilitate tree traversal, the header table is established and linked to the node where the data item appears in the tree for the first time [20].

The article "TCM Constitution Analysis Method Based on Parallel FP-Growth Algorithm in Hadoop Framework" was published in 2022. Journal: J Healthc Eng.

Then the process of frequent item set mining is realized through the FP-growth algorithm in the following steps: (i) Generate a conditional pattern base for a given suffix item. Firstly, find the set of leaf nodes IDs of the suffix item from the constructed FP-tree, and then start from each leaf node in the set, search the path from the leaf node to the root node recursively. All the combined paths of the set form the conditional pattern base of the given suffix. Especially, in the process of building the conditional pattern base of the given suffix, it is necessary to update the count that refers to the suffix item to accommodate the case of multiple leaf nodes superimposed. (ii) Frequency is determined based on the updated count of the item of conditional pattern base. FP-growth algorithm is a memory-based frequent pattern mining algorithm. Although FP-growth algorithm saves the scanning time and operational costs compared with the Apriori algorithm, it also is ineffective and memory-consuming when coping with massive clinical data to dig out its frequent patterns. What is more, the traditional multipoint interface (MPI) parallel programming model is facing the problems of node and network failures communication at the same time [21]. For the above two reasons, a new parallel programming framework is needed to satisfy the requirements of real clinical data mining.

### 2.2. Hadoop Framework

Hadoop is a famous distributed system infrastructure that allows users to develop distributed applications without knowing their underlying details and takes full advantage of the great power of clusters for reliable, efficient, and scalable computing and storage. Hadoop has been widely used in big data processing because of its natural advantages in data extraction, transformation, and loading (ETL). The distributed architecture of Hadoop keeps the big data processing engine as close to storage as possible, for example, ETL like batch operations can be directly oriented to storage.

Hadoop consists of many elements. At the lowest bottom is an open-source Hadoop distributed file system (HDFS), which stores files on all storage nodes in the Hadoop cluster. On top of HDFS is the MapReduce engine, which consists of JobTrackers and TaskTrackers two parts. Hadoop's MapReduce is a parallel computing framework that consists of two phases: Map and Reduce [22, 23]. In the Map phase, a single task is broken and these task pieces are sent to multiple nodes, which are then loaded into a data warehouse as a single data set in the reduce phase. The Map phase is responsible for the mapping of the data, also known as data transformation. The Reduce phase is responsible for the aggregation of data, which is important when looking for frequent item sets.

The article "TCM Constitution Analysis Method Based on Parallel FP-Growth Algorithm in Hadoop Framework" was published in 2022. Journal: J Healthc Eng.

MapReduce includes a job control module, programming model, and data processing engine. Here only the job control module is described in the following text. As the main control node of MapReduce, Master is mainly used to manage and execute scheduling tasks. As the slave node of Master, Worker is used to managing the computing tasks performed on each node. The Master node NameNode used for data storage and parallel computing can be set on either one node or different nodes [24]. The Worker nodes DataNodes used for data storage and parallel computing are combined to realize that each Worker processes the data stored in the local DataNode. The architecture diagram of Hadoop is shown in Figure 2.

In this article, frequent item sets for a transaction are obtained by accumulating the item sets in this TCM constitution database which is deployed on a distributed server based on Hadoop framework. The basic idea of clinical data decomposition is divide-and-conquer, that is, the whole clinical data for TCM constitution is divided into several subparts and stored in different server nodes. Fortunately, this step is implemented by Hadoop automatically and what needs to do is only just set the copy of transaction data in the database to the framework of the open-source HDFS. And then Hadoop framework will classify the clinical data and divide it into several blocks automatically. For each block, a copy is saved when the block is stored in an assigned node to avoid node loss caused by fault damage files [25, 26].

### 2.3. Distributed FP-Growth Algorithm

Since it is necessary to scan the entire transaction database, the computation speed of traditional association rules algorithms, whether Apriori or FP-growth, will decrease to a certain extent in the face of large amounts of distributed clinical data. Even though some researchers have put forward the method of multithreading to relieve the pressure of calculating experimental data, the memory of a single computer will become the bottleneck to limit the data volume to a certain level that FP-growth algorithm can cope with. It is well known that the most prominent advantage of Hadoop framework based on a cloud platform is its parallel processing capability. Therefore, in order to make the association rules algorithms can be better adapt to the requirements of large-scale data processing problems in various fields and take full use of big data technology, the distributed parallel processing capability of Hadoop is used to promote the accuracy and recall rates and reduce the time consumption in the process of data processing to a large extent. The whole framework of distributed FP-growth algorithm based on HDFS is shown in Figure 3.

The article "TCM Constitution Analysis Method Based on Parallel FP-Growth Algorithm in Hadoop Framework" was published in 2022. Journal: J Healthc Eng.

The basic idea of the improved FP-growth method is to search the local frequent item sets in a local FP-tree that is constructed in a local node of HDFS parallelly instead of generating a global FP-tree to mine the clinical data. The specific steps of the proposed algorithm are described in brief as follows:

- Step 1: Database sharding and parallel computing
- The local transaction database on each node of HDFS needs to be scanned twice in the improved FP-growth algorithm. In order to promote the scanning efficiency, the database is decomposed into several data sets, which are processed in parallel to obtain the local frequent 1-item set list for each data set at the first time scan. Here, the horizontal partitioning strategy is used for data set decomposition.
- Step 2: Generating the Local FP-tree
- The transactions in the local data sets are sorted for each node according to the frequent 1-item set. And then, a local FP-tree is constructed and mined. In the process of mining the frequent item set for a given transaction, it is not necessary to mine the data and information stored in other nodes. Therefore, there is no need to keep communication between nodes to save resources and time. At the end of this step, local frequent items are gained, especially, those local frequent items that do not meet the minimum support threshold will not be removed in this procedure.
- Step 3: Parallel FP-growth
- Each node of HDFS counts the frequency of data items of all data sets that are located in the right node and obtains the local frequent item set counts. Then the global frequency of each item is can be calculated through communication between each node and the nonfrequent items are deleted according to the minimum support threshold. Eventually, the global 1-item set of the whole database is acquired.
- Step 4: Aggregating to generate global FP-tree
- After the above steps, local frequent item sets will be transmitted to the Master node. Local FP-trees are traversed iteratively instead of generating a global FP-tree, and then a large number of conditional FP-trees are generated according to the frequent 1- item sets. In the end, the global frequent item sets can be gained through deleting those frequent items whose count and confidence of the support degree are not satisfied with the minimum threshold.

The article "TCM Constitution Analysis Method Based on Parallel FP-Growth Algorithm in Hadoop Framework" was published in 2022. Journal: J Healthc Eng.

In this article, the traditional association rules algorithm FP-growth in big data mining has been combined with the open-source HDFS in machine learning to promote the computation speed as far as possible to meet the requirements of solving the problem of TCM constitution automatic analysis. In the end, a classification model for TCM constitution was established to observe the accuracy of category prediction to provide preliminary screening and clinical decision support for physicians.

## 3. The Framework of ARA-TCM Algorithm

### 3.1. Algorithm Implementation Details

The proposed ARA-TCM algorithm for constitution analysis can be divided into four processes according to the execution order and function subject mentioned in abovementioned section. In the MapReduce programming framework of the Hadoop cluster, the proposed method is implemented in four steps: acquiring table chain, constructing local FP-tree, mining local frequent item sets, and searching the global frequent item set. Firstly, the data blocks in HDFS are read in parallel and the occurrence times of data items are counted to retain those data items that meet the minimum support threshold. Sort the remained data items in descending order of their counts of occurrences and insert the sorted data items into a chain table with a header. Secondly, each storage node in HDFS has a sorted header chain, which is easy to set up Map and Reduce functions to create a local FP-tree. Fortunately, it is the same way to build a local FP-tree through FP-growth algorithm by creating a chain table in Hadoop framework. Thirdly, mining a local frequent item sets of a local FP-tree is also similar to the way to mine a global FP-tree. Both of them delete the infrequent items according to the support and confidence degrees. Finally, the global frequency item sets are calculated through communication between each distributed node. What is more, in order to realize the parallel MapReduce model on the cloud platform to take full advantage of the high capability of Hadoop in processing big data, a method for producing frequent sets of *K* terms was proposed in this article, which is described in flow chart Figure 4.

As it is well known that in the theories of TCM, dietary regimens vary from person to person. That is, different symptoms collection corresponds to the different constitutions which has their unique health and conditioning schemes. Furthermore, dietary regimens of different people with the same constitution also can be different due to their individual differences such as ages, genders, health conditions, and so on. In other words, the relationships between individual symptoms and conditioning programs are so close that the dietary regimen should be carried out according to the individual symptoms. Therefore, training on the relationship between constitution and symptoms should be followed by training on constitution and health conditioning. This specific training process is mainly divided into two stages. The first stage is to perform two scans of the constitution data set to dig out the relationships of constitutions in relation to symptoms and health conditions, respectively, and the second stage is to link the symptoms, constitution, and dietary regimen.

The article "TCM Constitution Analysis Method Based on Parallel FP-Growth Algorithm in Hadoop Framework" was published in 2022. Journal: J Healthc Eng.

The specific algorithms for training on the relationships of constitutions in relation to symptoms and health conditions, respectively, are described as follows Algorithms 1 and 2, which are used to generate and mine the local frequent item sets, respectively.

Therefore, the whole searching process for the quantitative relationships between TCM symptoms and the feature vectors of physical analysis of clinical records is described as follows:

- Step 1: Input (line offset, physical symptom data training set *T*);
- Step 2: Output (symptom-1, constitution-1);
- Step 3: In the Map stage, output (symptom, constitution) for each symptom *I* in the physical characteristic data training set *T*;
- Step 4: In the Reduce phase, the sum of initialized frequent physical symptoms is 0. When value.hasNext counts, the sum is increased by 1. And then output (symptom, count) for each symptom *I*_*i*_ and its count number *N*_*i*_; at the end of this step, the occurrence times of data items are counted.
- Step 5: Input (line Offset, physical symptom data training set *T*);
- Step 6: Output (Prescription-1, Physical Fitness);
- Step 7: In the Map stage, *L* is equal to the sum of all the items of physical symptoms; And then data training set *T* is sorted in descending order Sort(prescription, constitution); Search the groupings of rightmost item sets of frequent item sets, if *Q*_*i*_ = seachGroup(t.get(t.length)- 1), print (*Q*_*i*_, 1);
- Step 8: In the Reduce phase, when FP is equal to LocalFPGrowth (symptom, Tree), output the occurrence count of the local frequent item (LocalFPcount, null);
- Step 9: In the processing stage, calculate the sum of all the item sets of physical symptoms. If FPcount is greater than the minimum support, output the frequent item FP and its occurrence number (FP, COUNT);
- Step 10: End of the algorithm.

The physical symptom data training set *T* that stored in the Hadoop platform was scanned in parallel for the first time. As mentioned above, a shorter scanning time will be acquired if parallelization is used to process the clinical TCM database. The constitution item with the highest occurrence frequency can be obtained after the first scan, which is recorded as constitution-1 and regarded as the header of the chain table. The frequency items whose occurrence counts are below the minimum support threshold will be deleted. The left constitution items are sorted in descending order of their count numbers to create a local FP-tree. In this article, the minimum support threshold is set to 20. This is because there are at least 20 symptom items according to the judging standards of the symptom physiques for TCM constitution analysis.

The article "TCM Constitution Analysis Method Based on Parallel FP-Growth Algorithm in Hadoop Framework" was published in 2022. Journal: J Healthc Eng.

Firstly, these constitutions with high occurrence frequency are divided into balanced groups. The group number is set to 9 because there are nine constitutions altogether in the theoretical system of TCM. The constitution-1 was divided into 9 groups according to the way of balanced grouping, and the constitution table with high occurrence frequency was obtained from these 9 groups. Secondly, the groupings of the rightmost item sets of 9 different constitutions are searched in Map phase. Then the packet number of each grouping is used as the primary key and the body is used as the value to transmit the grouping to the Reduce node by means of key value. In the Reduce phase, the local minimum support is screened according to the data items received in the Map phase, and a local FP-tree is generated on the basis of local minimum support. Thirdly, the local FP-tree is accessed in an ab initio table to obtain the conditional mode. The frequent constitutive item sets are mined by a recursive method based on the combination of multiple branching and single branching. After mining, the local frequent body item sets are stored in HDFS files. Finally, the global frequent constitution item sets were generated by merging all the local frequent constitution item sets. Here, the frequency constitution item sets in the HDFS file are obtained and added to local ones with the same frequent item to gain global support. In the end, the frequent constitution item sets whose overall supports are greater than the overall minimum support are retained and saved in an HDFS file.

The main task of the second stage is to link the symptoms, constitution, and regimen. As it has been mentioned in the above text, it is very important to find the relationships between symptoms and constitution, constitution, and health conditioning programs to TCM clinical diagnosis and treatment. Generally speaking, there are two ways to find this relationships. The first method is to put the training for physical symptoms and health conditioning programs into the Hadoop platform to find the correlations between them. The second approach is based on ontology rules between symptoms, TCM constitution, and dietary regimen since there are already known relationships between the three parameters which are obtained in the first stage.

The article "TCM Constitution Analysis Method Based on Parallel FP-Growth Algorithm in Hadoop Framework" was published in 2022. Journal: J Healthc Eng.

### 3.2. Algorithm Analysis

In this article, the data partitioning idea is combined with the working mechanism of Hadoop platform to simplify the flow of mining the TCM constitution frequent item sets. Compared with the classical FP-growth algorithm based on the distributed architecture of MapReduce, the proposed method has more advantages in data volume dispersion and load balancing. Unlike the traditional parallel FP-growth algorithm to generate a global FP-tree, there is no internode communication when generating and mining a local FP-tree on the node of HDFS. Therefore, the parallel FP-growth algorithm based on Hadoop not only has the advantages of shorter computation time and larger data processing capacity under the same amount of data but also solves the memory overflow problem of big data mining under certain conditions.

Usually, the time consumption of the distributed FP-growth algorithm is mainly divided into three parts: (1) counting the number of the data items to obtain the global support number and generating the header chain according to the support degree at the same time; (2) mining the local maximum frequent item set for each storage node; and (3) integrating the global maximum frequent item set that conforms the global support and confidence degrees both. The proposed ARA- TCM algorithm for TCM constitution analysis is based on HDFS. Supposing there are *n* storage nodes involved in the calculation, *p* Maps and Reduces can be processed simultaneously on each node, *q* transaction records in the entire database totally and *m* data items for each record on average. Then the time complexity of generating the header chain is *O*(*q*^*∗*^*m*/*n*_*∗*_*p*). Supposing *r* iterations are needed to mine the local maximum frequent item set for each storage node, then the time complexity of this process is *O*(*q*^*∗*^*m*^*∗*^*r*/*n*_*∗*_*p*). Finally, all the local frequent item sets are merged to find the global maximum frequent item set according to the support and confidence degrees together. Supposing the merged item set composes of *s* different frequent item sets, the time complexity is *O* (*s*). Especially, if the key of the local frequent item sets on *n* storage nodes are the same, the time complexity of the merging process is *O*(*s*/*n*). There is no need to communicate between nodes during the processes of generation and mining of local FP-trees. The larger number of Hadoop nodes and the more times of the MapReduce can be processed at a time, the lower time complexity and higher the implementation efficiency of the proposed algorithm.

The article "TCM Constitution Analysis Method Based on Parallel FP-Growth Algorithm in Hadoop Framework" was published in 2022. Journal: J Healthc Eng.

## 4. Experiment and Discussion

In this section, the proposed ARA-TCM algorithm for constitution analysis in Hadoop framework is evaluated on the following tasks. Especially, we want to determine:

- Can the proposed method reflect the TCM constitution patterns accurately?
- Can the proposed method find the rules between patients' constitution and effect of TCM herbs?
- Can the proposed ARA-TCM method achieve better precision and recall rates than other typical models?
- Can the proposed method reduce the training and actual losses dramatically?

In General, the proposed ARA-TCM method has been compared with typical Apriori and FP-growth algorithms. Both methods have been widely applied to data mining fields and achieved good results in reflecting the TCM constitution patterns and finding the treatment rules from the medical records. However, the proposed method has higher precision and recall rates, lower training, and actual losses comparing with Apriori algorithm.

### 4.1. Experimental Data Set

The medical records mainly come from Guangzhou Xiangxue Internet Hospital and classic medical records in history, which contain a large amount of reference medical cases. There are a total of 30,071 pieces of data, each piece of data represents a patient's complete diagnosis and treatment process, including the psychological and physiological symptoms, primary and secondary constitutions, treatment and medication plan, and so on.

In this work, these rec medical records are divided into 9 groups as it has been well known that there are 9 TCM constitutions, namely, balanced constitution (BC), yang-deficiency constitution (YADC), yin-deficiency constitution (YIDC), qi-deficiency constitution (QDC), qi-stagnation constitution (QSC), phlegm-dampness constitution (PDC), dampness-heat constitution (DHC), blood stasis constitution (BSC), inherited special constitution (ISC). At the same time, in order to make the experimental results are more robust and accurate, cross-validation method was used in this article. In the training process, the whole data is split into ten parts randomly. Nine parts were used as training samples and the left was used as test samples for each learning. And all ten test results were recorded to evaluate whether the average accuracy of ten test results meets expectations. If not, adjust the hyperparameters until optimal ones were obtained, and then, the whole data set is learned to achieve only the final expected model.

### 4.2. Experimental Implementation Details

The overall functional modules of TCM constitution analysis process are shown in Figure 5. And the specific implementation details for preliminary TCM constitution classification are described as follows.

(i) Step 1: Data Preprocessing
Noise filtering is the first necessary task before training module to make the learned model more accurate. A large number of literature mining data processing is required for the real clinical data before removing noisy symptom data. Therefore, preprocessing process can be divided into two stages: text processing and data noise removal. Generally speaking, the two types of preprocessing allow the continuous sentence in the text set to be represented as feature vectors, which are more suitable for constructing sample text data and subsequent word processing in the training process.
    Text processing stage: To avoid taking unnecessary words as features, it is a common way to descend the total number of entities by removing “irrelevant” words based on stops, these stagnation words usually include articles, auxiliary verbs, pronouns, prepositions, conjunctions and so on. For example, words such as “this,” “he/she/it,” “and,” and “or” occur frequently in the text are not able to distinguish or predict and can be removed from the input entities of the training module.
    Noise removing stage: Cluster method is used in this part. The noisy data refers to the same symptoms that will occur in different constitutions. Even if the number of the same symptoms is small, they should be removed to avoid the impact on the final results in the process of training. For instance, there is the same characteristic: pale red tongue for BC and QDC and this characteristic should be discarded when recognizing the two constitutions. Here clustering analysis was used to detect this kind of outliers by organizing similar features into groups (clusters). Intuitively, values that fall outside the cluster are considered outliers.
(ii) Step 2: Training module
The main aim of this step is to find out the correlation between constitution and physical symptoms. It has been known that each one corresponds to different physical features. The proposed ARA-TCM method was used to dig out the relationships between symptoms and physical rules based on the support and confidence of the association rules analysis method. Here “support” expresses the probability that a rule will occur and is used to measure the statistical characteristics of a rule; “confidence” represents the conditional probability that a rule will occur and is used to measure the accuracy of a rule. From Table 1, it can be found that the corresponding symptoms of a constitution are not single and only a combination of several symptoms with different weights of importance can accurately judge a certain constitution. Supposing “*A* <=> *B*” indicates an interaction between constitution *A* and symptom *B*. For example, *BC* <=> “complexion and moist skin color” means that one of the symptoms corresponding to *BC* is “complexion and ruddy skin color,” which will be regarded as a kind *o* expression that someone's constitution is balanced (BC).
(iii) Step 3: Constitution analysis module
The step is used to classify the obtained mining results in step 2. In the process of classification, it can be found that each kind of frequent item set of the constitution has its own representative frequent items of the physical symptoms, corresponding to the highest frequency of symptoms set, which is also known as the symptoms of frequent items.
(iv) Step 4: Testing module
In this step, some diseases were input into the learned TCM constitution analysis model to obtain the corresponding classification results for test. And then a reasonable regimen plan is recommended according to the analysis results.

The article "TCM Constitution Analysis Method Based on Parallel FP-Growth Algorithm in Hadoop Framework" was published in 2022. Journal: J Healthc Eng.

There are two things worth noting: (1) In the actual clinical syndrome differentiation, the collected data always suffers from low quality. That is not all of the information in the provided data set is useful for constitution analysis and health planning. Therefore, it is necessary to pre-process the input data set before sample training such as noise filtering, feature selecting, and so on to reduce the dimension, volume, and interference information of data to be trained. This operation is very crucial to shorten the training time and promote the classification accuracy and effectiveness for the finally TCM constitution analysis and health regimen recommendation results. (2) In the process of TCM constitution analysis, personal characteristics of a given patient are necessary to judge the types of patient's constitution to customize a reasonable health regimen based on individual physical health details. That is, even though there are nine types of constitution totally, doctors will also plan different health regimens for the people with the same constitution because of their gender, age, physical conditions, personal preferences, and so on under the guidance of the theory of TCM health theories. Therefore, the key to TCM constitution analysis is to grasp the main symptoms related to constitution identification directly, and distinguish the specific physical health status of patients clearly to make an accurate judgment.

### 4.3. Evaluation Methodology

Usually, classification precision rate *P*, recall rate *R,* and *F*-measure *F*1 are used to evaluate the experimental results and verify the ability of the proposed model to identify valuable data for TCM constitution analysis. Supposing TP and TN represent the numbers of true examples and false counterexamples, respectively, and TF and FN represent the false positive examples and true counterexamples, respectively. And AIR = TP + FN represents the total number of samples truly related to TCM constitution in the whole test data set, CDR = TP + TN is regarded as the number of data records that are consistent with their actual categories during the data training and DR = TP + FP represents the number of samples that the constructed models found from the whole test data. Therefore, these criteria for model evaluation can be defined as follows:

(1) $$\begin{array}{c} P=\frac{TP}{DR}\\ =\frac{TP}{TP+FP}\times 100\%,\\ R=\frac{TP}{\text{AIR}}\\ =\frac{TP}{TP+FN}\times 100\%,\\ F_{1}={\left(\frac{R^{-1}+p^{-1}}{2}\right)}^{-1}\\ =2\frac{P\cdot R}{P+R}. \end{array}$$

*F*1 value is the harmonic mean of precision and recall rate. The errors between the real result and the predicted results of the training set and testing set, respectively, refer to the training loss and actual loss of the model. In order to make the experimental results of feature training and prediction more stable and robust, cross-validation method was used to acquire the average values of the above criteria. In this article, the entire clinical data set was divided into ten subsets randomly. Nine subsets were regarded as training sample sets and the left one was used as the test sample set to obtain the values of precision rate, recall rate, and *F*-measure. After 10 rounds of training and testing, the average values of the criteria were obtained. *F*1 value

The article "TCM Constitution Analysis Method Based on Parallel FP-Growth Algorithm in Hadoop Framework" was published in 2022. Journal: J Healthc Eng.

### 4.4. Experimental Results

#### 4.4.1. TCM Constitution Analysis

In this work, the proposed method was used to explore the association rules between the 9 kinds of TCM constitutions and symptoms, as well as the regimen treatment plans to discover the rules of typical clinical symptoms and treatment rules of different constitutions and to conduct evidence-based medical evaluation of TCM effects in the constitution-related chronic disease health management. In the end, a knowledge set “disease symptoms constitutions treatments/regimen” was conducted during the training process and it is found that the top three constitutions are mid constitution (42.3%), hot and humid constitution (31.3%), and inherited special constitution (26.2%), respectively. Rules of typical symptoms for each constitution contained in the specific data set of “symptoms constitution” are shown in Table 1. The rules of constitutions between diseases and drugs are also studied in this work. Here, phlegm-dampness constitution (PDC) is taken as an example to show the excavated results between constitution, diseases, and drugs.

The article "TCM Constitution Analysis Method Based on Parallel FP-Growth Algorithm in Hadoop Framework" was published in 2022. Journal: J Healthc Eng.

There are 13 kinds of diseases are related to PDC. The top 5 diseases are The top five diseases were hypertension, nonalcoholic fatty liver disease, obesity/overweight, dyslipidemia, and type 2 diabetes, which are mainly chronic diseases. Basically, it can be concluded that diseases related to PDC are mainly cardiovascular and metabolic diseases, among which, cardiovascular diseases are mainly hypertension, and metabolic diseases are mainly abnormal blood lipid/glucose and obesity. In view of these chronic diseases, TCM prescriptions are mainly used to improve physical constitution with the overall guiding principle to eliminate phlegm and remove dampness. In this work, It is mainly focused on Chinese medicinal drugs.

There are more than 300 kinds of drugs used to treat PDC-involved diseases in the medical records and 30 kinds of drugs are used more than 3 times in TCM prescriptions. According to the theory of “Chinese materia medica,” the 30 drugs can be classified as tonifying deficiency drugs, invigorating water and permeating dampness drugs, reducing phlegm, relieving cough and antiasthmatic drugs, promoting blood circulation and removing stasis drugs, reducing dampness drugs, relieving surface drugs, clearing heat drugs, closing astringency drugs, regulating qi drugs, calming liver and dispelling wind drugs, appetizing and eliminating food drugs and purging medicine. The most frequently used drugs were tonics for deficiency, including atractylodes, Chinese yam, licorice root, and white lentil beans. The second is water infiltration medicine, including tuckahoe, coix seed, and Alisma; then the antitussive pinellia; Salvia miltiorrhiza is the main medicine for promoting blood circulation and removing blood stasis. Dehumidification medicine is atractylodes bark, and magnolia bark; the remedies are Pueraria root and vegetable household. Antipyretics include rhizoma coptidis and cassia seed. These drugs belong to the spleen meridian, lung meridian, stomach meridian, and liver meridian, which also shows that the clinical treatment of PDC is to follow the theory of traditional Chinese medicine.

#### 4.4.2. Evaluation Parameters

As can be seen from Table 2, the proposed ARA-TCM method based on FP-growth algorithm in Hadoop framework has higher recognition precision and recall rates than Apriori algorithm in TCM constitution analysis field. The average recall rate is above 53% and the average precision rate is above 85%, which means the proposed method is able to identify the samples related to TCM constitution more effectively. Apriori algorithm and FP-growth algorithm are very classical and have been widely applied in mining association rules inner data. The proposed ARA-TCM is constructed based on FP-growth algorithm and HDFS in Hadoop framework to cope with massive distributed medical data. Therefore, comparative experiments were conducted with the three methods mentioned above to classify TCM constitution under the same simulation environment and good results have been obtained. The time consumed by the three methods for processing the same amount of clinical data is shown in Figure 6. As mentioned above, the experimental clinical data comes from Guangzhou Xiangxue Internet Hospital, containing a total of 30,071 pieces of data. The random sampling method was used in the experiments to obtain data sets of different volumes.

The article "TCM Constitution Analysis Method Based on Parallel FP-Growth Algorithm in Hadoop Framework" was published in 2022. Journal: J Healthc Eng.

In the field of information retrieval and natural language processing, precision rate, recall rate, and comprehensive evaluation index *F*1-measure are three important parameters to judge the quality of models. Especially in medical data mining, it is crucial to find the right information as much as possible to avoid misdiagnosis. In this article, precision rates and recall rates acquired by the three methods for comparison with the three methods under the same numbers of samples are shown in Figures 7 and 8, respectively. Training losses of the related training data sets and the actual loss of the relevant test sets acquired by the three methods for comparison with three methods for comparison are shown in Figures 9 and 10, respectively. Finally, *F*1 measures are shown in Figure 11 to evaluate the overall state of each method.

From Figure 9, it can be found that ARA-TCM method has a lower loss rate than Apriori and FP-Growth algorithms after the training stage with various data sets of different volumes. And what is more, the training loss is gradually reduced with the gradual increase of the volume of data sets and trends to be stable finally, which means that association rules algorithms are better suited for handling data sets with large volumes. The errors obtained by the proposed method are also lower than those acquired by the other two algorithms in the testing processes for TCM constitution analysis. It has been proved that the ARA-TCM method performs a little bit better in terms of accuracy. In terms of the overall situation *F*1 of the three algorithms in TCM constitution analysis, although the ARA-TCM algorithm was lower than the FP-growth algorithm at the beginning, the overall situation in the later period was relatively in line with expectations, which means the proposed method is more suitable for processing large volume data and consistent with characteristics of HDFS.

The article "TCM Constitution Analysis Method Based on Parallel FP-Growth Algorithm in Hadoop Framework" was published in 2022. Journal: J Healthc Eng.

Whether assuming symptoms used for TCM constitution analysis to be independent of each other or making Apriori algorithm start from the quantitative relationship between constitution categories and symptoms, is very impractical in the actual clinical TCM constitution identification. Therefore, it is carried out by calculating the prior probability and class-conditional probability to realize the TCM constitution classification. However, when the occurrence frequency of some symptoms is very low in an unbalanced data set, the sparsity problem is likely to occur and the probability calculated will be very small, resulting in relatively a large deviation of results in the actual classification prediction process. But in fact, the proposed ARA-TCM method can avoid this problem be-cause its distributed processing model for training in Hadoop framework. According to the physical symptoms and their corresponding optimal parameters of prescription, the physical type can be calculated and predicted. The proposed ARA-TCM method predicts that there is a 42.3% probability of being mild constitution (BC), 31.3% probability of being hot and humid (DHC), and 26.2% probability of being a special constitution (ISC). Although such prediction may have some deviations, it can undoubtedly provide important decision support for TCM physique analysis. In addition, because the training set given may belong to different constitutions simultaneously, the proposed method based on FP-growth algorithm and HDFS is more suitable for multicategory recognition than Apriori algorithm. Therefore, ARR-TCM method can be more and adapted for TCM constitution analysis.

## 5. Conclusion and Future Work

In this article, an improved association rules algorithm (ARA-TCM) based on FP-growth algorithm in Hadoop framework has been proposed for TCM constitution analysis and regimen recommendation, which is able to acquire better experimental results with higher precision and recall rates in comparison to the classical Apriori algorithm. However, there is still room left for improvement in the future TCM constitution recognition and analysis. Inquiring about symptoms in the clinical data set involves a lot of subjective feelings from patients such as painful, energetic, fatigued, excessive sweating, and so on. In other words, the TCM constitution identification results will be affected by the patients'subjective feelings, resulting inaccurate diagnosis. A better solution would be adding tongue image and pulse signal on the basis of inquiring symptoms to discover more accurate knowledge for TCM constitution analysis in data mining process to make the proposed method more suitable for this specific application.

The article "TCM Constitution Analysis Method Based on Parallel FP-Growth Algorithm in Hadoop Framework" was published in 2022. Journal: J Healthc Eng.

## Figures and Tables

**Figure 1:** Flow chart of FP-growth algorithm.

**Figure 2:** Hadoop framework diagram.

**Figure 3:** Flow chart of distributed FP-growth based on Hadoop.

**Figure 4:** The process of producing frequent sets of *K* terms.

**Figure 5:** Flow chart for preliminary classification process of TCM constitution.

**Figure 6:** Consumption of time.

**Figure 7:** Comparison of precision rates.

**Figure 8:** Comparison of recall rates.

**Figure 9:** Comparison of training loss.

**Figure 10:** Comparison of actual loss.

**Figure 11:** Comparison of *F*1.

**Algorithm 1:** Generating local frequent item sets.

**Algorithm 2:** Mining local frequent item sets with FP-growth.

**Table 1:** Constitutions with typical corresponding symptoms.

Constitution typic	Typical symptoms
Balanced (BC)	Pale red tongue thin white moss ruddy complexion dense and shiny hair energetic…
Yang-deficiency (YADC)	Fat and tender tongue dark lips black eyes think hair fat and soft muscle chilly…
Yin-deficiency (YIDC)	Red tongue thin flushed face dry mouth and throat pulse breakdown…
Qi-deficiency (QDC)	Pale red tongue pulse weak fat or thin pale face easy fatigue…
Qi-stagnation (QSC)	Unstable introversion sensitive and anxious depressed insomniac…
Phlegm-dampness (PDC)	Sticky mouth and greasy moss oil and sweet skin somnolent and lethargic fat and soft belly edema eyes…
Dampness-heat (DHC)	Easily upset and irritable lethargic prone to acne and acne fat or thin…
Blood stasis (BSC)	Blue and purple lip rough and dark skin black eyes irritability and forgetfulness easy itchy and achy yellow hair…
Inherited special (ISC)	Prone to be allergic. Poor immunity easy to urticaria easy to allergic rhinitis easy to asthma easy to skin desquamation…

**Table 2:** Computational results.

Model	AIR	DR	TP	*P* (%)	*R* (%)
Apriori	1890	921	639	69.38	48.73
ARA-TCM	1890	1172	996	84.98	62.01

## Data Availability

No data were used to support this study.
